# Lamin B2 promotes the progression of triple negative breast cancer via mediating cell proliferation and apoptosis

This article has been retracted.

**DOI:** 10.1042/BSR20203874

**Published:** 2021-01-29

**Authors:** Cui-Cui Zhao, Jing Chen, Li-Ying Zhang, Hong Liu, Chuan-Gui Zhang, Yan Liu

**Affiliations:** 1 Department of VIP Ward, Tianjin Medical University Cancer Institute and Hospital, Tianjin, P.R. China; 2 National Clinical Research Center for Cancer, Tianjin’s Clinical Research Center for Cancer, Key Laboratory of Cancer Prevention and Therapy, Tianjin, P.R. China; 3 Key Laboratory of Breast Cancer Prevention and Therapy, Tianjin Medical University, Ministry of Education, Tianjin, P.R. China; 4 Department of Pancreatic Oncology, Tianjin Medical University Cancer Institute and Hospital, Tianjin, P.R. China; 5 Department of internal medicine, Mudanjiang Cancer Hospital, Mudanjiang, P.R. China; 6 Second Department of Breast Surgery, Tianjin Medical University Cancer Institute and Hospital, Tianjin, P.R. China

**Keywords:** Apoptosis, Breast cancer, Lamin B2 (LMNB2), Proliferation, Target, Triple negative breast cancer (TNBC)

## Abstract

Triple negative breast cancer (TNBC) is a more common type of breast cancer with high distant metastasis and poor prognosis. The potential role of lamins in cancer progression has been widely revealed. However, the function of lamin B2 (LMNB2) in TNBC progression is still unclear. The present study aimed to investigate the role of LMNB2 in TNBC. The cancer genome atlas (TCGA) database analysis and immunohistochemistry (IHC) were performed to examine LMNB2 expression levels. LMNB2 short hairpin RNA plasmid or lentivirus was used to deplete the expression of LMNB2 in human TNBC cell lines including MDA-MB-468 and MDA-MB-231. Alterations in cell proliferation and apoptosis *in vitro* and the nude mouse tumorigenicity assay *in vivo* were subsequently analyzed. The human TNBC tissues shown high expression of LMNB2 according to the bioinformation analysis and IHC assays. LMNB2 expression was correlated with the clinical pathological features of TNBC patients, including pTNM stage and lymph node metastasis. Through *in vitro and in vivo* assays, we confirmed LMNB2 depletion suppressed the proliferation and induced the apoptosis of TNBC cells, and inhibited tumor growth of TNBC cells in mice, with the decrease in Ki67 expression or the increase in caspase-3 expression. In conclusion, LMNB2 may promote TNBC progression and could serve as a potential therapeutic target for TNBC treatment.

## Introduction

Breast cancer is one of the most common cancers and fatal diseases in the world [1]. Approximately 10–20% of breast cancers are triple negative breast cancer (TNBC) [2]. Compared with other types of breast cancer, TNBC have three common features, including more invasive, higher grade, and a ‘basal-like’ cell type [3]. The prognosis of TNBC is worse than other types of breast cancer [4]. Currently, the traditional treatment method for TNBC patients is mastectomy combined with chemotherapy and radiotherapy [1,5]. Despite atezolizumab and nab-paclitaxel have been approved for programmed death ligand 1-positive metastatic TNBC, there are still several unsolved problems in immunotherapy of TNBC [6]. Recently, the great prospect of targeted therapy for TNBC has been noticed [7]. However, in order to improve the prognosis of TNBC patients, identification of new therapeutic targets for precise treatment of TNBC is still badly needed.

Lamin proteins play significant roles in nuclear stability, chromatin structure maintenance, and gene expression regulation [8–10]. Vertebrate lamins consist of two types, A and B [11]. Lamin B (LMNB) has two isoforms, including LMNB1 and LMNB2 [12]. According to previous literature reports, in different tumors, the expression levels of LMNB1 and LMNB2 are different, and their effects on tumor development are also different, so targeted studies are needed [12]. LMNB2 is involved in a variety of critical physiological and pathological processes [13–15]. Previous study showed that mutations of genes in *lamin* family might cause acquired partial lipodystrophy and myoclonus epilepsy with early ataxia [15,16].

Recently, the potential roles of lamins in cancer progression have been widely revealed [17,18]. LMNB1 expression has been found correlated with poor prognosis of patients with hepatocellular carcinoma (HCC) [19], cervical cancer [20], and colon cancer [21]. LMNB2 had significant relationship to non-small cell lung cancer (NSCLC) [22]. However, the potential role of LMNB2 in TNBC progression is still unclear.

Herein, we designed the present study and found LMNB2 could serve as a promising therapeutic target for the treatment of TNBC. The high expression of LMNB2 in human TNBC tissues was found by cancer genome atlas (TCGA) database analysis and immunohistochemistry (IHC) assays. High expression of LMNB2 was correlated to a more malignant clinicopathological status. LMNB2 depletion suppressed the proliferation and induced the apoptosis of TNBC cells *in vitro*, and inhibited tumor growth of TNBC cells in mice. Our findings therefore indicated the potential role of LMNB2 in TNBC progression.

## Materials and methods

### Tissue specimens

A total of 82 TNBC specimens in this study were surgical specimens with complete clinicopathological data collected in our hospital. All studies were approved by our Ethics Committee. Informed consent was obtained from all patients.

### Antibodies

The following antibodies were used for immunoblot and immunohistochemistry assays: LMNB2 (Abcam, ab151735, 1:1000 dilution for immunoblot, 1: 100 dilution for immunohistochemistry), β-actin (Abcam, ab8226, 1:1000 dilution), Ki67 (Abcam, ab16667, 1:1000 dilution), and Caspase-3 (Abcam, ab2302, 1:500 dilution).

### IHC assays

The sections of 4 μm thickness were prepared on charged glass slides. After deparaffinization and rehydration, slides were immersed in 10 mM citrate buffer (pH = 7.5) and microwaved at 750 W for 30 min for antigen retrieval. Endogenous peroxidase activity was blocked by adding 3% hydrogen peroxide. The sections were subsequently incubated with diluted antibodies followed by polymerconjugated horseradish peroxidase in a humidified chamber. Standard diaminobezidin staining was performed for chromogenic detection of the IHC targets.

The score method was briefly described as follows. The proportion of positive staining cells: 0, negative tumor cells or < 10% positive tumor cells; 1 means 10–50% positive tumor cells, and 2 means > 50% positive staining cells. The staining intensity was assessed on a score of 0 (negative staining), 1 (modest staining), or 2 (strong staining). LMNB2 expression levels were calculated according to the staining scores: staining intensity score + positive tumor cell staining score. Staining scores 0, 1, and 2 were considered LMNB2 low-expression, when 3 and 4 were LMNB2 high expression.

### Cell culture and transfection

The TNBC cell lines MDA-MB-468 and MDA-MB-231 were purchased from the American type culture collection (ATCC, Manassas, VA, U.S.A.). These types of cell lines were maintained in Dulbecco’s modified eagle medium (DMEM, Gibco, Waltham, MA, U.S.A.) and supplemented with 10% fetal bovine serum (FBS, Gibco), 100 ng/ml streptomycin and 100 U/ml penicillin (Gibco). Cells were incubated at 37°C with 5% CO_2_. Transfection of these two cell lines was performed using Lipofectamine 2000, according to the manufacturers’ instructions. For an example, in six-well plates, 5 μl transfection reagent and 2 μg short hairpin RNA (shRNA) plasmids were mixed in 500 µl serum-free DMEM, left to stand for 5 min and then mixed. After incubation at room temperature for 20 min, the mix was added to serum-starved cells and incubated at 37°C for 4 h. For the control group, the shRNA targeting sequence was nonsense and did not target intracellular RNAs. Target sequence for LMNB2 shRNA used in this study was GGCTGCAGGAGAAGGAGGAGCTG.

### RNA isolation and quantitative polymerase chain reaction (qPCR) assays

The levels of LMNB2 mRNA were detected with qPCR assays. Total RNA was isolated from cells using Trizol reagent (Invitrogen, Waltham, MA, U.S.A.) and used for the first strand cDNA synthesis with the reverse transcription system (Roche, Indianapolis, IN, U.S.A.) following the manufacturer’s protocol. The following thermocycling conditions were used for qPCR: initial denaturation at 95°C for 3 min; followed by 30 cycles of denaturation at 95°C for 30 s, annealing at 58°C for 30 s, and extension at 72°C for 30 s. The 2-ΔΔCq method was used to quantify the results. GAPDH was used as a loading control. Primer sequences: GAPDH, forward 5′-CGACCACTTTGTCAAGCTCA-3′ and reverse 5′-GGTTGAGCACAGGGTACTTTATT-3′; LMNB2, forward 5′-AGAAGTCCTCGGTGATGCGTGA-3′ and reverse 5′-CATCACGTAGCAGCCTCTTGAG-3′.

### Immunoblot assays

The breast cancer cells were washed by phosphate buffer saline (PBS) buffer and subsequently lysed with radio immunoprecipitation assay buffer (50 mM Tris-HCl/pH 7.4; 1% NP-40; 150 mM NaCl; 1 mM ethylene diamine tetraacetic acid; 1 mM proteinase inhibitor; 1 mM Na_3_VO_4_; 1 mM NaF; 1 mM okadaic acid; and 1 mg/ml aprotinin, leupeptin, and pepstatin). The BCA method was used for protein determination. Proteins (20 µg/lane) were separated on 8% sodium dodecyl sulfate polyacrylamide gel electrophoresis gel and transferred onto polyvinylidene fluoride (PVDF) membranes on the ice (250 mA, 2 h). Subsequently, the membranes were blocked with 5% dry milk in Tris buffered saline Tween (TBST) buffer for 2 h and incubated with antibodies, and washed with TBST buffer. Then PVDF membranes were developed in electrochemical luminescence mixture and visualized by Imager.

### Colony formation assays

Approximately 1000 cells were seeded in six-well plate with three replicates. The culture medium was replaced with 2 ml fresh medium every 2 days. After 4 weeks, colonies were fixed with paraformaldehyde for 30 min at room temperature, stained with 0.2% Crystal Violet for 30 min, and then photographed and counted manually.

### Flow cytometry detection of apoptosis

TNBC cells were collected, centrifuged, washed with PBS, then resuspended in 100 μl of binding buffer with 5 μl of annexin V—fluorescein isothiocyanate, and incubated at room temperature for 10 min. Subsequently, 5 μl of propidium iodide solution was added and the cells were incubated for another 5 min at room temperature. Apoptosis cells were detected and analyzed by a flow cytometer (Beckman Coulter, Brea, CA).

### *In vivo* xenograft assays

Sterilized Balb/c nude mice (female, 5 weeks old, 14–16 g) were provided by Beijing Vital River Laboratory Animal Technology Co., Ltd. (Beijing, China), fed with food and water ad libitum, and kept at a specific pathogen-free level at 20°C and a humidity of 60%, alternating between light and dark for 12 h. None of the mice died accidentally during the study. The mice were killed by cervical dislocation, and their heartbeat was checked to determine whether they were dead, on the last day of the experiment. The mice were randomly divided into two groups (5 mice per group) and treated with control or LMNB2 stably depleted MDA-MB-231 cells. About 5 × 10^6^ cells were injected subcutaneously into nude mice. The volume of the tumor was measured every 3 days using a vernier caliper from the 15th day after injection. The tumor volume was calculated as follows: Tumor volume (mm^3^) = Tumor length (mm) × Tumor width (mm)^2^ / 2.

### Statistical analysis

GraphPad 5.0 software was used for statistical analysis in the present study. All experiments were carried out three times, and all results were represented as mean ± standard deviation (Mean ± SD). The Kaplan–Meier curve analysis method was conducted for the survival analysis. The correlation was calculated using Fisher’s exact test and χ2 analysis. Student’s *t*-test was used for statistical comparisons. * indicates *P*<0.05, which was considered a statistically significant difference.

## Results

### LMNB2 expression is enhanced in human TNBC cancer tissues

To explore the role of LMNB2 in TNBC progression, the LMNB2 expression levels were first compared between 1085 tumor tissues and 291 normal tissues according to TCGA database. We found LMNB2 was high expression in human TNBC tissues (*P*<0.05, Figure 1A). Meanwhile, LMNB2 expression was significantly correlated to disease-free survival rates of patients with TNBC in different groups (Figure 1B,C), suggesting that LMNB2 affected the prognosis of TNBC patients. Subsequently, the expression of LMNB2 was assessed in TNBC tissues and the corresponding normal tissues via IHC staining. As shown in Figure 2, the LMNB2 expression was abnormally increased in human TNBC tumor tissues compared with the normal tissues.

**Figure 1:** Bio-analysis revealed that LMNB2 was highly expressed in TNBC tissues and correlated with the prognosis of TNBC patients (**A**) The TCGA database showed the expression levels of LMNB2 in tumor tissues and the corresponding normal tissues. (**B** and **C**) The TCGA database exhibited the correlation between LMNB2 and disease-free survival rates in TNBC patients from different case groups. *P<0.05.

**Figure 2:** LMNB2 was high expression in human TNBC tissues (**A**) IHC assays were performed to detect LMNB2 expression in human TNBC tissues, and the representative photographs were shown (100× and 200× magnification, respectively). (**B**) The results of IHC assays exhibited the expression levels of LMNB2 in corresponding normal tissues (H&E stain, 100× and 200× magnifications, respectively).

### High expression of LMNB2 was correlated to poor clinicopathologic features of TNBC patients

Based on the staining levels of LMNB2 in tumor tissues, TNBC patients were divided into two groups, including low LMNB2 expression group (*n*=30, 36.6%) and high LMNB2 expression group (*n*=52, 63.4%). The expression of LMNB2 in TNBC tissues was correlated with clinical pathological characteristics, including pTNM stage (*P*=0.036) and lymph node metastasis (*P*=0.034, Table 1). However, no significant correlation was found between LMNB2 expression and age, tumor grade, and tumor size (Table 1).

**Table 1:** Relationships of LMNB2 and clinicopathological characteristic in 82 patients with TNBC

Feature	All (*n*=82)	LMNB2 expression		χ^2^	*P*
		Low (*n*=30)	High (*n*=52)		
Age (years)				3.577	0.059
<55	48	14	34		
≥55	34	16	18		
Tumor grade			2.395	0.122	
Low	50	15	35		
High	32	15	17		
Tumor size			0.216	0.642	
<2	52	20	32		
≥2	30	10	20		
pTNM stage			4.389	0.036*	
I-II	60	26	34		
III-IV	22	4	18		
Lymph node metastasis			4.518	0.034*	
No	42	20	22		
Yes	40	10	30		

* *P*<0.05.

### LMNB2 was effectively down-regulated in TNBC cells caused by the transfection of LMNB2 shRNA plasmid

The levels of LMNB2 mRNA were significantly reduced in MDA-MB-468 and MDA-MB-231 cells transfected with LMNB2 shRNA plasmids, those were confirmed by qPCR assays (Figure 3A). Meanwhile, the protein levels of LMNB2 were also down-regulated in LMNB2 shRNA-transfected MDA-MB-468 and MDA-MB-231 cells by immunoblot assays, those were consistent with the results of qPCR assays (Figure 3B).

**Figure 3:** LMNB2 expression was effectively reduced in both MDA-MB-468 and MDA-MB-231 cells after the transfection of its shRNA plasmids (**A**) qPCR assays exhibited the effective decrease expression of LMNB2 after the transfection of its shRNA plasmids in MDA-MB-468 and MDA-MB-231 cells, respectively. (**B**) Immunoblot assays exhibited the obvious decrease of LMNB2 expression levels following the transfection of its shRNA in MDA-MB-468 and MDA-MB-231 cells. Results are presented as mean ± SD, * *P*<0.05.

### Knockdown of LMNB2 has anti-proliferation effects on TNBC cells *in vitro*

The ablation of LMNB2 dramatically suppressed the proliferation of MDA-MB-468 and MDA-MB-231 cells, with the obvious decrease in colony number (Figure 4A). Consistent with the results of colony formation assays, LMNB2 depletion also significantly blocked the expression of Ki67 in MDA-MB-468 and MDA-MB-231 cells, which was confirmed by immunoblot assays (Figure 4B).

**Figure 4:** LMNB2 promotes cell proliferation of TNBC *in vitro* LMNB2 promotes cell proliferation of TNBC *in vitro*. (**A**) Colony formation assays were performed in MDA-MB-468 and MDA-MB-231 cells upon the transfection of control or LMNB2 shRNA plasmids, and the number of colonies was manually counted. (**B**) Immunoblot assays exhibited the expression levels of Ki67 in the transfection of control or LMNB2 shRNA plasmids in MDA-MB-468 and MDA-MB-231 cells. *P<0.05

### LMNB2 depletion induced the apoptosis of TNBC cells

The results of flow cytometry assays showed ablation significantly stimulated the apoptosis of MDA-MB-468 and MDA-MB-231 cells, with the increased proportion of apoptosis cells (Figure 5A,B). The expression levels of caspase-3 were dramatically increased, caused by the depletion of LMNB2 in MDA-MB-468 and MDA-MB-231 cells (Figure 5C).

**Figure 5:** LMNB2 depletion stimulated the apoptosis of TNBC cells *in vitro* (**A** and **B**) Flow cytometry assays were performed in MDA-MB-468 and MDA-MB-231 cells transfected with control or LMNB2 shRNA plasmids, and the proportion of apoptosis cells was compared between control and LMNB2 depletion cells. (**C**) Immunoblot assays exhibited the expression levels of caspase-3 in MDA-MB-468 and MDA-MB-231 cells transfected with control or LMNB2 shRNA plasmids. Results are presented as mean ± SD, * *P*<0.05.

### LMNB2 contributes to tumor growth of TNBC cells in mice

LMNB2 shRNA lentivirus was used to stably deplete LMNB2 expression in MDA-MB-231 cells. Then the control or LMNB2 ablation cells were injected into nude mice, respectively. After 15 days, we isolated tumors and measured the volume of tumors every 3 days. The tumor volumes following LMNB2 depletion were obviously smaller those of the control group (Figure 6A). IHC assays further confirmed LMNB2 expression levels in tumors from LMNB2-depletion group were obviously decreased compared to the control group (Figure 6B). In accordance with the previous *in vitro* data, the expression of Ki67 in tumor tissues was decreased after LMNB2 depletion, whereas the caspase-3 expression was obviously increased (Figure 6C,D).

**Figure 6:** LMNB2 contributes to tumor growth of TNBC cells in mice (**A**) MDA-MB-231 cells infected with control or LMNB2 shRNA lentivirus were subcutaneously implanted into nude mice. After 15 days, the tumors were isolated and photographed, and the tumor volumes were measured every 3 days. Tumor growth curves were calculated and compared between LMNB2 knockdown and control groups. IHC assays showed the expression levels of LMNB2 (**B**), Ki67 (**C**), and caspase-3 (**D**) in tumors of the control or LMNB2 depletion groups. Results are presented as mean ± SD, * *P*<0.05.

## Discussion

Breast cancer is one of the most fatal diseases for women in the worldwide [1]. TNBC has the worst prognosis among all breast cancer subtypes [2]. It is characterized by high rate of visceral metastasis, easy recurrence, and low survival rate [4]. Combing surgical operation with radiotherapy and chemotherapy are currently the primary reliable therapeutic options for TNBC patients, whereas these treatments could not cure the patients exactly [5]. Therefore, novel and effective therapeutic targets and precise treatment hold great promise to combat TNBC. Several therapeutic targets, such as polyadenosine diphosphate ribose polymerase and vascular endothelial growth factor (VEGF), have been studied for many years and have the potential to develop as targeted therapy drugs for TNBC [23].

Many researchers have identified multiple specific molecular targets those can be used for TNBC cancer therapy, such as intra-nuclear targets, intracellular targets, cell surface targets, and immune checkpoint modulators [24,25]. Recently, the potential role of lamins in the progression of different cancers has been widely revealed [17,18]. LMNB2 is a nuclear lamin protein and may be one of the intra-nuclear targets [12]. It was reported that microRNA-122 inhibits HCC cell progression via targeting LMNB2 [26]. LMNB2 was also found to be significantly related with NSCLC progression [22]. However, the role of LMNB2 in TNBC progression is still unclear. In the present study, we revealed LMNB2 could serve as a novel molecular target for TNBC treatment.

First, bioinformation analysis results suggested that LMNB2 was highly expressed in breast invasive carcinoma and correlated with the prognosis of TNBC. In our study, we demonstrated that LMNB2 in tumor tissues of TNBC patients in China have higher expression than that in normal tissues by IHC. LMNB2 expression was also correlated with the clinical pathological features including pTNM stage and lymph node metastasis.

This is different from other types of lamin proteins. The expression of LMNB1 was negatively associated with pTNM stage, tumor grade, and clinical outcome [27]. The function of lamin A/C is similar to that of LMNB1. Reduced or loss of expression of lamin A/C was related to the worse prognosis and shorter outcome in early-stage breast cancer [28]. Similarly, high lamin B2 expression correlated with shorter overall survival of NSCLC patients [22]. Therefore, among these lamin proteins, LMNB2 is the most likely therapeutic target for the treatment of breast cancer. As B-type lamins are constitutively expressed in most cell types, it may be necessary to improve drug targeting by local administration or nanodelivery for TNBC treatment.

Subsequently, the effects of LMNB2 on TNBC cell proliferation and apoptosis were investigated *in vitro*. LMNB2 was effectively down-regulated upon the transfection of LMNB2 shRNA plasmid in TNBC cells. Depletion of LMNB2 inhibited the proliferation by blocking the expression of Ki67, and induced apoptosis process of TNBC cells by increasing caspase-3 expression. This is consistent with that LMNB2 can promote the proliferation, migration, and invasion of HCC cells [26].

We also explored the effect of LMNB2 depletion on tumor growth of TNBC cells in mice. As was expected, the tumor volumes of mice in LMNB2-depletion group were smaller than those of control groups, and the expression of LMNB2 and Ki67 in tumor tissues of LMNB2-depletion mice were conspicuous decreased, while caspase-3 expression was increased, compared to that of the control mice. This may suggest that LMNB2 can inhibit TNBC tumor growth in mice by decreasing ki67 expression and increasing caspase-3 expression. As we know, Ki67 and caspase-3 played irreplaceable role in the TNBC cells proliferation and apoptosis, which are related to multiple signaling pathways, such as PI3K/AKT, RAS/RAF/ERK [29].

However, the precise molecular mechanism and the signaling pathway underlying LMNB2 regulating TNBC tumor growth are still unclear and needs to be further investigated. Previous reports showed that microRNA-122 inhibited HCC cell progression via targeting LMNB2 [26] and confered sorafenib resistance to HCC cells by RAS/RAF/ERK signaling pathway [30]. LMNB2 may affect the development of HCC and breast cancer through RAS/RAF/ERK signaling pathway. Signaling pathways related to LMNB2 and TNBC tumor development are also worth further study.

In summary, our results suggested that the expression of LMNB2 in tumor tissues of TNBC patients was higher than that in adjacent tissues. High LMNB2 expression was correlated with a more malignant clinicopathological status of TNBC patients. LMNB2 depletion suppressed the proliferation, induced the apoptosis of TNBC cells *in vitro*, and inhibited tumor growth of TNBC cells *in vivo*. LMNB2 may therefore be a potential therapeutic target for the development of new drugs and the treatment of TNBC.

## Data Availability

The datasets generated and analyzed during the current study are available from the corresponding author on reasonable request.

## Abbreviations

IHC: immunohistochemistry
HCC: hepatocellular carcinoma
LMNB2: lamin B2
NSCLC: non-small cell lung cancer
TCGA: The cancer genome atlas
TNBC: triple negative breast cancer
